The article "Fitness Promotion in a Jump Rope-Based Homework Intervention for Middle School Students: A Randomized Controlled Trial" was published in 2022. Journal: Front Psychol.

# Fitness Promotion in a Jump Rope-Based Homework Intervention for Middle School Students: A Randomized Controlled Trial

**DOI:** 10.3389/fpsyg.2022.912635

**Published:** 2022-06-16

**Authors:** Fang Huang, Ying Song, Yingdong Zhao, Yating Han, Qun Fang

**Affiliations:** ^1^School of Physical Education, Qingdao University, Qingdao, China; ^2^School of Physical Education, Shandong University, Jinan, China; ^3^Department of Physical Education and Sport Science, Mudanjiang Medical University, Mudanjiang, China

**Keywords:** adolescents, homework, jump rope, physical activity, fitness promotion

## Abstract

Physical activity (PA) homework offers a promising approach for students to be physically active after school. The current study aims to provide holistic insights into PA homework design and the effects of implementation in practice. In total, ninety-three middle school students were randomly assigned to a homework group (HG) or control group (CG). Participants in HG (*n* = 47) were requested to complete jump rope homework three times per week for 12 weeks, while their counterparts in CG attended one health education class every week. A homework sheet was used to provide instructions and record information for exercise behaviors during homework completion. Physical fitness tests were conducted to investigate the effects of the jump rope homework on the physical fitness of middle school students. After the intervention, participants in HG reported moderate to vigorous PA during jump rope exercise. The average duration for each practice was approximately 48 min. The returned homework sheets accounted for 86.88% of all homework assignments, indicating a good completion rate. Compared with their counterparts in CG, participants performing jump rope exercise indicated greater improvement in speed, endurance, power, and core muscular endurance. Jump rope homework strengthened physical fitness for middle school students, which provided a valuable addition to comprehensive school PA practice.

## Introduction

Inadequate physical activity (PA) increases the risks of chronic diseases (i.e., obesity and cardiovascular disease) among children and adolescents, which has raised global public health concerns (Hills et al., 2011; Landry and Driscoll, 2012; Gupta et al., 2013). A recent study reported that over 80% of adolescents worldwide failed to meet the daily moderate-to-vigorous physical activity (MVPA) recommendations [Bull et al., 2020; Guthold et al., 2020; World Health Organization [WHO], 2020]. Regular PA has been considered necessary in weight control and obesity-related disease prevention (Poitras et al., 2016; Brown et al., 2019). A physically active lifestyle in childhood and adolescence often continues into adulthood and improves overall well-being at an older age (Landry and Driscoll, 2012; McPhee et al., 2016). In addition to the health-related considerations, the development of motor skills provides another reason for PA engagement during childhood and adolescence. The neuromuscular system is highly plastic during critical periods, which imply an optimal time for developing motor skills (Gabbard, 2012). Missing the critical period for a specific function makes it difficult to reach full potential in adult life (Salkind, 2002; Gale et al., 2004). Therefore, the developmental perspective also highlights the importance of achieving adequate PA levels at a young age.

School plays a critical role in influencing students’ daily PA level because of accessible resources for PA participation, such as sports facilities and competent physical educators (Pate et al., 2000; Trost et al., 2008). In addition, a large number of children and adolescents spend most of their daytime at school (Ha et al., 2015; Baumgartner et al., 2020). Therefore, the school has been considered an ideal setting for PA intervention (Story et al., 2009). However, due to the increasing demand for academic achievement, PA levels tend to decline as students age, which poses challenges in school health practice (Pate et al., 2002; Dumith et al., 2011; Rauner et al., 2015). As an extension of school-based PE programs, PA homework addresses the already limited and still-shrinking time for PA participation at school (Mitchell et al., 2000a). Time spent after school is characterized by a high level of sedentary behaviors (Trost et al., 2008). Making good use of this time period has the potential to increase daily PA for children and adolescents (Naylor et al., 2008; Duncan et al., 2011, 2019). Indeed, after-school PA programs have been proved effective in decreasing the risk of obesity (Martínez Vizcaíno et al., 2008), developing motor and cognitive functions (Kamijo et al., 2011), improving academic performance (Durlak et al., 2010), and leading to physically active lifestyles (Lee et al., 2020).

Jump rope is a whole-body movement that allows participants to engage in MVPA. Average metabolic equivalent (MET) was reported to reach 11.7 and 12.5 in a 5-min rope skipping at a rate of 125 reps/min and 145 reps/min, respectively (Ainsworth et al., 2000). Consistent findings were identified in another study using the OMNI perceived exertion scale and heart rate as measures of exercise intensity. The OMNI scale is a category rating format that contains both pictorial and verbal descriptors positioned along a numerical response range of 0–10 (Robertson et al., 2000). Children (aged 10.6 ± 0.9 years) reported an average score of 6.4 and a corresponding heart rate of 180 bpm when skipping at the rate of 140 reps/min. The results suggest moderate to high-physical exertion during the jump rope exercise (Buchheit et al., 2014).

The specific advantages of jump rope make it a promising exercise modality within and beyond school settings. Jump rope is characterized by low requirements for physical space and equipment cost, which facilitate access to PA (Ha et al., 2014). Schools, particularly in Asian countries, are usually crowded with a large number of students (Johns and Ha, 1999). A feasible solution to the space restrictions would be of great value in practice. Jump rope can be performed in limited space, which justifies its wide application to school-based PA (Hao et al., 2019; Baumgartner et al., 2020). Affordability is another advantage of jump rope, which addresses PA barriers related to low socioeconomic status (Kim et al., 2020; Yang et al., 2020). Students from lower socioeconomic areas face an increased risk of obesity (Stamatakis et al., 2010). Affordable equipment is regarded as a critical factor in encouraging PA and lowering relevant health risks in this population (Ha et al., 2015, 2017). Motivation is a key factor in PA participation and adherence over time (Yang and Xu, 2014). Research has shown that participants would be more motivated if exercise was perceived as fun (Kim et al., 2020). Jump rope is considered an enjoyable exercise modality for adolescents (Hernandez et al., 2009; Ha et al., 2014; Sung et al., 2019; Yang et al., 2020), which implies the feasible application of jump rope to PA homework.

In the existing research, homework was mainly delivered through non-active forms such as sports event attendance, written assignments (Mitchell et al., 2000b), and fitness concept learning (Jorgenson and George, 2001). The effects of active homework on physical fitness largely remain unknown. Claxton and Wells (2009) conducted a 12-week PA homework program among college students. Based on self-reported PA levels, the study indicated that homework could be an effective method of increasing the PA of college students. The study design can be further improved in two aspects. First, the subjective survey can be replaced by an objective assessment. Second, while homework has been proved effective in PA promotion, further investigations can focus on the influence of homework on physical fitness. The current study aims to provide holistic insights into PA homework design and the effects of implementation in practice. It is our interest to investigate whether homework assigned in the form of jump rope could improve physical fitness for middle school students.

## Materials and Methods

### Study Design and Recruitment

A two-arm parallel group RCT was conducted following the Consolidated Standards of Reporting Trials (CONSORTs) (Boutron et al., 2008). The study consisted of the following four phases: recruitment, pre-test, intervention, and post-test. Recruitment was conducted in the first 2 weeks of the spring semester (March) in 2021. All the participants were recruited from a middle school in Qingdao, China. Research assistants answered questions from the students and parents to ensure research information to be fully acknowledged. Eligible participants should meet the following criteria: (1) participants and their parents signed the informed consent forms; (2) participants were not student athletes; (3) participants had no recent injury that impaired motor performance; and (4) participants did not attend any other after-school PA programs during the study.

The eligible participants were randomly assigned to either a homework group (HG) or a control group (CG). All the participants completed the pre-test in the 3rd week of the semester. The 12-week intervention was then conducted from weeks 4 to 15. Different tasks were assigned to HG and CG during the intervention. Participants in HG completed jump rope homework, while their counterparts in CG attended health education classes. The post-test was conducted in the 16th week of the semester (July).

The recruitment initially identified 116 students who expressed their willingness to participate in the study. The screening process excluded 23 students because of regular participation in after-school PA programs (*N* = 12), student athletes (*N* = 10), and recent injury (*N* = 1). Therefore, 93 eligible participants (men = 46, women = 47) were randomly assigned to HG (*N* = 47, women = 24) or CG (*N* = 46, women = 23). A one-way independent ANOVA was conducted to compare HG with CG at the baseline. No significant between-group differences were identified in age, body mass index (BMI), or measures of physical fitness (Table 1). Figure 1 displays the enrollment and allocation processes. The study was conducted in accordance with the Declaration of Helsinki and approved by the Ethics Committee of Qingdao University.

**TABLE 1:** Statistics of one-way independent ANOVA.

	HG (*n* = 47)	CG (*n* = 46)	*p*-value
Age (year)	14.43 ± 0.62	14.37 ± 0.64	0.67
BMI (kg/m^2^)	19.08 ± 2.03	19.53 ± 2.39	0.32
Broad jump (m)	1.77 ± 0.27	1.80 ± 0.25	0.47
50 m sprint (s)	8.94 ± 0.62	9.02 ± 0.64	0.57
Sit-up	33.26 ± 4.37	32.57 ± 5.73	0.52
Sit-and-reach (cm)	13.28 ± 4.32	13.40 ± 4.83	0.90
800 m run (s)	222.70 ± 34.98	219.09 ± 27.65	0.58

*HG, homework group; CG, control group; BMI, body mass index.*

**FIGURE 1:** Flow diagram of enrollment, allocation, follow-up, and data analysis.

### Randomization and Blinding

Participants were assigned a computer-generated number before allocation. Another set of numbers was randomly generated by the computer to identify the participants allocated to HG. Allocation was carried out by an external researcher for the consideration of concealment. Researchers were blinded because there was no direct interaction between researchers and participants. While the participants in HG completed the assigned homework, those in CG attended health classes led by a hired instructor who was not involved in any part of the research. It is worth noting that participant blinding may be somewhat compromised in the current study. Participants were blinded only if they were unable to distinguish between treatments applied to different groups (Maher et al., 2003). Because all the participants were at the same school, the current design could not exclude the possibility that participants of HG and CG might realize the different treatments during daily communication.

### Intervention

The participants in CG attended health classes every Friday from 5:10 to 5:50 p.m. The class was instructed by a specialist in health education. Knowledge on nutrition, exercise, and a healthy lifestyle was provided. On the other hand, participants in HG completed a 45-min jump rope exercise every Monday, Wednesday, and Friday during after-school hours (after 5 p.m.). In total, eight fundamental skipping drills were selected, including basic hop, alternate foot step, scissors, front-and-back jumps, side-to-side jumps, “jumping jack,” single leg jumps, and double under. The drills were introduced and practiced in the first 15 min of each PE class as warm-up activities. Because all the students had experience of learning and practicing jump rope in elementary school, the skipping drills were familiar to the participants.

To facilitate homework completion, we designed a homework sheet (Figure 2) that listed the workout plan with detailed information as to drills for practice, skipping rate, the number of sets, and break time. The sheet also had blanks for participants to report the date of exercise, start time, practice duration, and rating of perceived exertion (RPE). The participants were asked to turn in the completed homework sheet and received a new one from research assistants. The homework was recommended rather than required, as participants and their parents acknowledged that the homework completion did not influence their final grade in physical education.

**FIGURE 2:** Example of homework sheet for participants in HG.

Trusting students to complete their PA homework honestly is an issue faced by PE teachers and researchers (Gabbei and Hamrick, 2001). The current study adopted strategies to hold students accountable for the completion of homework. Participants needed to turn in the completed homework sheet to their PE teachers in exchange for a new one for the next practice. To enhance parental involvement, we asked parents to sign the sheet as a verification that the participants completed the practice as suggested (Gabbei and Hamrick, 2001; Hart, 2001). The homework sheet was valid only if it was completely filled out and signed by parents.

### Descriptive Statistics of Homework Completion

Descriptive statistics were collected to reflect homework completion. The percentage of valid homework sheets received from the participants indicated the rate of homework completion. Start time and duration provided information for the homework implementation. RPE has been shown to be a valid and convenient instrument to quantify the intensity of exercise and training (Foster et al., 2001; Impellizzeri et al., 2004). The Borg Category-Ratio (CR) scale was used to measure the exercise intensity of perceived effort (Shariat et al., 2018). Participants reported a score between 0 (no effort at all) and 10 (maximal effort) to reflect physical exertion during the jump rope homework.

### Measures of Physical Fitness

Physical fitness was assessed by five tests on speed, flexibility, core muscular endurance, explosive power, and endurance. Speed was measured by a 50 m sprint. Time was automatically recorded by an infrared system with a precision of 0.01 s (Model: CSTF–FH, Tongfang Co., Ltd., China). Students started in a standing position. The better performance in two trials was recorded. Flexibility was assessed by a sit-and-reach test. Participants slowly reached as far as possible with one hand on top of the other and keeping their knees straight on the floor. Performance was measured by an electronic device with a precision of 0.1 cm (Model: CSTF–YW, Tongfang Co., Ltd., China). Participants conducted two trials in the sit-and-reach test. The longer distance was used as the measure of flexibility performance. Explosive power was assessed by broad jumping. The electronic device (Model: CSTF–TY, Tongfang Co., Ltd., China) automatically recorded the jump distance with the precision of 0.1 cm. Two attempts were allowed in the test, and the better performance was used for data analysis. Sit-ups have been shown to be effective for measuring core muscular endurance for both male and female (Bianco et al., 2015). Participants lie on a cushion with their knees bent at approximately right angles. Participants placed one hand over the other on the chest, and raised their body toward their knees. Successful repetitions in 1 min were counted by trained research assistants. Endurance was assessed by an 800 m run on a standard 400-m lap. Research assistants used stopwatches to record the times of participants completing the test. Participants performed once in both the sit-up test and 800 m run.

### Statistical Analysis

Data analysis was performed in two steps. First, one-way repeated measures ANOVA was used for pre- and post-test comparisons of each individual group. The independent variable consisted of two time intervals: pre- and post-test. Dependent variables were the outcomes of the fitness tests on speed, flexibility, core muscular endurance, explosive power, and endurance. Second, a 2 × 2 repeated measures multivariate analysis of variance (MANOVA) was conducted to investigate the effects of jump rope homework on physical fitness, with group (HG and CG) as a between-group factor and time (pre-test and post-test) as a within-group factor. Outliers were defined as 3 SDs from the mean. The Shapiro–Wilk test was performed to verify the normality assumption. The homogeneity of variance assumption was checked by Levene’s test of equality of error variances. The effect size was calculated by partial eta squared (η^2^), with values of 0.01, 0.06, and 0.14 defining small, moderate, and large effects (Cohen, 1988). Statistical significance was defined by the cutoff point of 0.05. All the statistical analyses were conducted by SPSS 25.

## Results

The 47 participants performing jump rope homework were supposed to submit 1,692 homework sheets in 36 sessions throughout the 12-week intervention. A total of 1,470 valid homework sheets were received by the end of the intervention, which accounted for 86.88% of all homework assignments. The distribution of the start time showed that most practices (19.09%) began between 8:00 p.m. and 8:30 p.m. Over 70% of practices began after 7:00 p.m., indicating that a majority of participants were available for PA during the time period (Figure 3). Jump rope homework took 47.98 (SD = 6.87) minutes on average, which was longer than the scheduled 45-min practice (*t*_*46*_ = 2.97, *p* = 0.01). Participants reported a mean RPE score of 5.28 (SD = 1.95), suggesting a moderate to vigorous level of PA associated with jump rope homework.

**FIGURE 3:** Distribution of time participants began jump rope exercise.

Participants in HG showed significant improvement in broad jump (*F*_1,46_ = 372.56, *p* < 0.001, η^2^ = 0.89), 50 m sprint (*F*_1,46_ = 17.16, *p* < 0.001, η^2^ = 0.27), sit-up (*F*_1,46_ = 50.24, *p* < 0.001, η^2^ = 0.52), and 800 m run (*F*_1,46_ = 39.53, *p* < 0.001, η^2^ = 0.46), but not in sit-and-reach (*F*_1,46_ = 0.13, *p* = 0.73, η^2^ = 0.003). In addition, participants in CG indicated significant improvement in broad jump (*F*_1,45_ = 25.03, *p* < 0.001, η^2^ = 0.36), sit-up (*F*_1,45_ = 14.79, *p* < 0.001, η^2^ = 0.25), and 800 m run (*F*_1,45_ = 10.60, *p* = 0.002, η^2^ = 0.19). But there was no significant change in 50 m sprint (*F*_1,45_ = 2.26, *p* = 0.14, η^2^ = 0.05), or sit-and-reach (*F*_1,45_ = 0.26, *p* = 0.61, η^2^ = 0.01). The results of the one-way repeated measures ANOVA are summarized in Table 2.

**TABLE 2:** Statistics of one-way repeated measures ANOVA by individual groups.

Tests	Groups	Pre-test	Post-test	Change score	*p*-value
Broad jump (m)	HG	1.77 ± 0.27	1.97 ± 0.24	0.20 ± 0.07	*p* < 0.001
	CG	1.80 ± 0.25	1.87 ± 0.23	0.07 ± 0.09	*p* < 0.001
50 m sprint (s)	HG	8.94 ± 0.62	8.84 ± 0.56	−0.10 ± 0.17	*p* < 0.001
	CG	9.02 ± 0.64	8.99 ± 0.61	−0.03 ± 0.13	*p* = 0.14
Sit-up	HG	33.26 ± 4.37	37.15 ± 4.22	3.89 ± 3.77	*p* < 0.001
	CG	32.57 ± 5.73	33.96 ± 5.69	1.39 ± 2.45	*p* < 0.001
Sit-and-reach (cm)	HG	13.28 ± 4.32	13.10 ± 5.10	−0.18 ± 3.47	*p* = 0.73
	CG	13.40 ± 4.83	13.15 ± 6.31	−0.25 ± 3.28	*p* = 0.61
800 m run (s)	HG	222.70 ± 34.98	213.34 ± 31.12	−9.36 ± 10.21	*p* < 0.001
	CG	219.09 ± 27.65	215.83 ± 28.38	−3.26 ± 6.79	*p* = 0.002

*HG, homework group; CG, control group.*

The repeated measures MANOVA identified significant time by group interaction effects in broad jump (broad jump: *F*_1,91_ = 61.59, *p* < 0.001, η^2^ = 0.40), 50 m sprint (*F*_1,91_ = 5.46, *p* = 0.02, η^2^ = 0.06), sit-up (*F*_1,91_ = 14.35, *p* < 0.001, η^2^ = 0.14), and 800 m run (*F*_1,91_ = 11.46, *p* = 0.001, η^2^ = 0.11), suggesting a significant difference in performance change between HG and CG. Further analysis on change scores indicated greater improvement in HG than CG, which provided evidence for the favorable effects of jump rope intervention on the physical fitness. In addition, a significant main effect of time was also identified in broad jump (broad jump: *F*_1,91_ = 249.39, *p* < 0.001, η^2^ = 0.73), 50 m sprint (*F*_1,91_ = 17.46, *p* < 0.001, η^2^ = 0.16), sit-up (*F*_1,91_ = 63.99, *p* < 0.001, η^2^ = 0.41), and 800 m run (*F*_1,91_ = 49.07, *p* < 0.001, η^2^ = 0.35), indicating improved performance over time. HG and CG showed comparable performance given the fact that the main effect of group was non-significant in all measures of physical fitness. Jump rope exercise indicated limited impact on flexibility because of the non-significant results in the main effect of time (*F*_1,91_ = 0.37, *p* = 0.054, η^2^ = 0.004), main effect of group (*F*_1,91_ = 0.01, *p* = 0.93, η^2^ = 0.001), and time by group interaction effect (*F*_1,91_ = 0.01, *p* = 0.092, η^2^ < 0.001). Table 3 indicates statistics of the repeated measures MANOVA.

**TABLE 3:** Statistics of the repeated measures MANOVA.

Tests	Time effect	Group effect	Interaction effect
Broad jump (m)	*F*_1,91_ = 294.39	*F*_1,91_ = 0.35	*F*_1,91_ = 61.59
	*p* < 0.001	*p* = 0.56	*p* < 0.001
	η^2^ = 0.73	η^2^ = 0.004	η^2^ = 0.40
50 m sprint (s)	*F*_1,91_ = 17.46	*F*_1,91_ = 0.78	*F*_1,91_ = 5.46
	*p* < 0.001	*p* = 0.38	*p* = 0.02
	η^2^ = 0.16	η^2^ = 0.01	η^2^ = 0.06
Sit-up	*F*_1,91_ = 63.99	*F*_1,91_ = 0.06	*F*_1,91_ = 14.35
	*p* < 0.001	*p* = 0.06	*p* < 0.001
	η^2^ = 0.41	η^2^ = 0.04	η^2^ = 0.14
Sit-and-reach (cm)	*F*_1,91_ = 0.37	*F*_1,91_ = 0.01	*F*_1,91_ = 0.01
	*p* = 0.54	*p* = 0.93	*p* = 0.92
	η^2^ = 0.004	η^2^ = 0.001	η^2^ < 0.001
800 m run (s)	*F*_1,91_ = 49.07	*F*_1,91_ = 0.01	*F*_1,91_ = 11.46
	*p* < 0.001	*p* = 0.93	*p* = 0.001
	η^2^ = 0.35	η^2^ < 0.001	η^2^ = 0.11

## Discussion

The current study implemented a 12-week PA homework intervention by means of jump rope exercise. Participants reported engaging in MVPA during homework completion. The participants might be undergoing a growth spurt during adolescence, which was evident by the improved physical fitness in CG. It is worth pointing out that participants in HG showed greater improvement than their counterparts in CG. The repeated measures MANOVA indicated significant interaction effects on speed, endurance, power, and core muscular endurance, suggesting additional benefits of jump rope exercise for the pubertal growth. The findings also indicate an integration of multiple elements into jump rope exercise (Pangrazi and Beighle, 2010; Trecroci et al., 2015). Concurrent development in agility, coordination, balance, and reaction can be achieved by means of variations in rope swing, skipping drills, movement directions, and stepping rhythms (Orhan, 2013; Partavi, 2013; Eler and Acar, 2018; Yang et al., 2020). In addition, the quick stretch-shortening cycle contractions during repetitive jumps indicate the characteristics of plyometric training which has been proved effective in improving speed and jump performance (Miyaguchi et al., 2014; García-Pinillos et al., 2020). It is worth noting the limited effects of jump rope exercise on flexibility. A practical implication is that stretching practice is needed after jump rope exercise for flexibility improvement.

Over the past decade, the Comprehensive School Physical Activity Program (CSPAP) has been widely accepted and applied to school health practice. The idea of CSPAP is to provide students with adequate PA opportunities by means of a multi-component approach before, during, and after school hours (Pulling Kuhn et al., 2021). Quality PE is the foundation of the program, along with the other four components, namely, PA during school, PA before and after school, family and community engagement, and staff involvement (Erwin et al., 2013). However, research has shown a limited effect of school-based PA interventions on the physical fitness and health behaviors of students. Love et al. (2019) conducted a meta-analysis on 17 studies. Evidence showed that school-based PA programs did not positively impact students’ physical activity. Therefore, implementing PA homework during after-school hours is an important addition to school PE. Yang et al. (2020) conducted a jump rope-based intervention program during after-school hours (5:00 p.m. to 6:00 p.m.). Jump rope classes were guided by instructors and conducted in a school gym. Significant improvement in muscular strength, body composition, and bone mineral density was identified in the jump rope group compared with the control group. In the current study, participants conducted the jump rope homework in a self-regulated approach. Although the amount of PA can be warranted in a well-organized, instructor-led jump rope class, implementing such an intervention program imposes a high level of demand on resources within the school (i.e., quality instructors and well-equipped facilities). Jump rope homework, on the other hand, does not require particular facilities and resources for PA participation, thus indicating prominent potential for wide applications.

The current study explored strategies to implement an effective PA homework program. Mitchell et al. (2000b) summarized four essential factors for successful homework, including relevance of homework to class content, understanding of homework, parent support, and student accountability. In fact, the jump rope homework was designed and implemented in compliance with the factors proposed in the previous study. To ensure all participants in HG completed the homework, PE teachers used the first 15 min of each class to teach the skipping drills assigned to the homework. Jump rope is considered ideal to warm-up activities because it is more active and dynamic than traditional routines of stretching and jogging (Chu, 1998). By integrating jump rope into the warm-up section of PE classes, we established a connection between homework and class content. Printed learning materials have been proved a useful instrument in administering homework (Weston et al., 1997; Gabbei and Hamrick, 2001). In the current study, the homework sheet provided explicit instructions on the drills, skipping rate, the number of sets, and break time. It has been noticed that the importance of clear task descriptions for homework completion (Gabbei and Hamrick, 2001). The instructions provided in the homework sheet facilitated participants’ understandings of practice. Parental involvement is another determinant of homework completion (Smith and Claxton, 2003). We asked parents to verify children’s performances and efforts by signing the homework sheet. The signature involved parents with the responsibility of assistance and supervision, which has been considered a useful strategy to hold students accountable for homework completion (Hart, 2001).

It is also important to stress the positive role of jump rope in facilitating access to PA after school. Evidence shows that over 70% of practices begin after 7 p.m. Because the students usually left school at 5 p.m., it might take time for the commute, dinner, and homework for other subjects. In fact, choosing jump rope as the homework content was based on a series of practical considerations. When designing the homework intervention, we realized the likelihood that students might do the homework at night. Compared with popular sports such as soccer and basketball, jump rope is suitable to play at night. To organize a team sport, specific requirements on court, lighting, and the number of participants need to be counted. A homework based on team sport might not be completed if any of the conditions were not satisfied. Jump rope addresses restrictions in time and space. Such advantages in organization and implementation enabled participants to do exercise when they were available. The percentage of valid homework suggests jump rope is feasible for PA homework.

To our knowledge, this is the first study applying the randomized controlled design to investigate the effects of active homework on physical fitness for middle school students. The empirical evidence contributed to in-depth understandings of PA homework design and implementation. However, the limitations of the current study must be clarified. The PA homework enhanced the physical fitness of the participants, but the long-term effects of the intervention were unclear. A follow-up test would be helpful to examine the sustainability of the program, which should be addressed in future studies. Another concern with the current study design lies in the lack of control over participants’ exercise behaviors throughout the study. Attending the health education classes could have led the students of CG to increase their PA level, which might eventually affect the differences between groups in physical fitness. In addition, because all participants were recruited from the same school, it is possible that participants in CG might actually take part in the intervention with their friends assigned to HG. Parental role in homework completion should be considered as well. Although previous research assumed a positive role of parents in stimulating students’ PA participation (Gabbei and Hamrick, 2001; Hart, 2001), it is necessary to raise awareness of the situation in which parents and participants in HG could easily fake good compliance. The limitation in study design could lead to a contamination of the results. In the current study, statistical analyses indicated significant differences in the magnitude of improvement between groups. It is reasonable to assume that either participants in CG taking part in jump rope exercise or faking good compliance with the PA homework would decrease the between-group differences in physical fitness. The significant difference between HG and CG suggests a limited impact of those behaviors, if any, on the findings. Lacking effective methods of evaluating participants’ exercise behaviors at home is a major challenge in both research and teaching practice, which needs to be addressed in the subsequent research to ensure successful completion of PA homework.

## Conclusion

The current study investigated the effects of a 12-week jump rope homework intervention on the physical fitness of middle school students. Participants reported MVPA in the jump rope exercise and showed a good completion rate of the homework. Jump rope exercise induced significant improvements in speed, endurance, power, and core muscular endurance. Further comparisons between groups indicated greater improvement in speed, endurance, power, and core muscular endurance of participants in HG, indicating additional jump rope benefits for pubertal growth. The promising findings on exercise behaviors and physical fitness lead to the conclusion that PA homework based on jump rope exercise is effective in enhancing physical fitness for middle school students.

## Data Availability Statement

The raw data supporting the conclusions of this article will be made available by the authors, without undue reservation.

## Ethics Statement

The studies involving human participants were reviewed and approved by Ethics Committee of Qingdao University. Written informed consent to participate in this study was provided by the participants’ legal guardian/next of kin.

## Author Contributions

FH and YH: conceptualization and writing—original draft preparation. FH and QF: methodology. YS and YZ: validation. FH and YS: formal analysis. QF, YZ, and YS: writing—review and editing. YZ: visualization. YH and QF: supervision. YH: project administration. All authors collaborated in preparing the manuscript.

## Conflict of Interest

The authors declare that the research was conducted in the absence of any commercial or financial relationships that could be construed as a potential conflict of interest.

## Publisher’s Note

All claims expressed in this article are solely those of the authors and do not necessarily represent those of their affiliated organizations, or those of the publisher, the editors and the reviewers. Any product that may be evaluated in this article, or claim that may be made by its manufacturer, is not guaranteed or endorsed by the publisher.
